# *In vitro* and *in vivo* responses of macrophages to magnesium-doped titanium

This article has been retracted.

**DOI:** 10.1038/srep42707

**Published:** 2017-02-15

**Authors:** Bin Li, Huiliang Cao, Yaochao Zhao, Mengqi Cheng, Hui Qin, Tao Cheng, Yan Hu, Xianlong Zhang, Xuanyong Liu

**Affiliations:** 1 Department of Orthopedics, Shanghai Sixth People’s Hospital, Shanghai Jiao Tong University, Shanghai 200233, China; 2 State Key Laboratory of High Performance Ceramics and Superfine Microstructure, Shanghai Institute of Ceramics, Chinese Academy of Sciences, Shanghai 200050, China

## Abstract

Modulating immune response to biomaterials through changing macrophage polarization has been proven to be a promising strategy to elicit beneficial outcomes in tissue repair. The objective of this study was to evaluate the response of macrophage polarization to titanium doped with magnesium (0.1~0.35%), which was prepared through the magnesium plasma immersion ion implantation (Mg PIII) technique. The M1/M2 polarization profile of macrophages was investigated using a murine cell line RAW 264.7 *in vitro* and a murine air pouch model *in vivo*. Our results demonstrated that the Mg PIII-treated titanium induced a higher percentage of M2 macrophages and higher concentrations of the anti-inflammatory cytokines interleukin (IL)-4 and IL-10. Genes encoding two growth factors, bone morphogenetic protein 2 (BMP2) and vascular endothelial growth factor (VEGF) were up-regulated, thus indicating the ability of the M2 phenotype to promote wound healing. The nuclear factor κB (NF-κB) signalling pathway was down-regulated. *In vivo* the Mg PIII -treated titanium elicited a similar effect on macrophage polarization and induced thinner fibrous capsule formation and a decrease in infiltrated cells. These results indicate that Mg PIII treatment has the immunomodulatory potential to elicit the pro-healing M2-polarized macrophage phenotype, thus providing new insight into the development of immunomodulatory biomaterials.

Titanium and its alloys are commonly used in implantable medical devices because of their good biocompatibility and desirable physical properties, such as their low modulus, good corrosion resistance, and high fatigue strength^1^. However, the undesirable inflammation caused by the implant itself and injuries following the surgical procedure of implantation have limited further applications^2^. This post-implantation inflammation leads to granulation tissue development, foreign body reactions, and fibrous capsule formation, all of which impair tissue regeneration and integration between the adjacent tissue and implants and may even cause implant failure^3^,^4^. Thus, it is essential to develop strategies to down-regulate the inflammatory response of the host and to elicit beneficial healing processes, thereby prolonging the life-span of titanium implants^5^.

Macrophages play a critical role in host reactions after the insertion of biomaterials. Macrophages are highly plastic, and their phenotypes and functions change in response to various environmental cues. According to their different biological functions, activated macrophages can be divided into two groups: M1, the “classically activated” pro-inflammatory macrophages, and M2, the “alternatively activated” anti-inflammatory macrophages. The M1 macrophages produce mediators such as IL-6, tumour necrosis factor (TNF)-α, inducible nitric oxide synthase (iNOS), and interferon (IFN)-γ, thereby promoting inflammation. The M2 macrophages express anti-inflammatory cytokines such as IL-4, IL-10, and arginase-1 (ARG) and consequently promote the resolution of inflammation and the regeneration of tissue^6^. Macrophage phenotypes and functions are highly relevant to biomaterial surface characteristics such as surface chemistry, pore size, strain and topography^7^. Regulation of the response of macrophage polarization to biomaterials provides intriguing strategies to elicit beneficial outcomes^8^,^9^,^10^,^11^. Magnesium (Mg), the second-most abundant divalent cation in cellular systems, plays important roles in the immune system, in both the innate and acquired immune responses, also known as the nonspecific and specific immune responses^12^. Mg also exerts an anti-inflammatory effect that is used clinically for multiple purposes, for instance, in obstetrics to treat seizure prophylaxis^13^. However, the high dose of magnesium (60 mg/L or 2.5 mM) used clinically via systemic administration raises the concerns about hypermagnesaemia^14^. This complication can result in a high risk of mortality by affecting the cardiovascular system and respiratory system^15^,^16^. Thus, local delivery of magnesium might be a better option to avoid affecting the anti-inflammatory activity.

Plasma immersion ion implantation (PIII), a non-line-of-light technique (in which the path of propagation of energetic doping atoms is not obscured by obstacles) for surface doping, may be a good pathway for local delivery of magnesium onto implantable medical devices. Previously, Mg PIII-treated titanium has demonstrated good osteogenic properties mediated by local release of Mg ions^17^,^18^. However, less is known about the immunomodulatory effects of Mg PIII treatment. Accordingly, in this study, we investigated the effect of Mg PIII-treated titanium on macrophage polarization *in vitro* and *in vivo*.

## Results

### Material characterization

The surface morphologies of the samples were observed by scanning electron microscopy (SEM). There were no obvious differences in the microstructures among the four groups (Ti, Mg30, Mg90, and Mg120), as shown in Fig. 1a. X-ray photoelectron spectroscopy (XPS) was used to reveal the chemical states of the surface components. The content of magnesium loading increased from 0.1% to 0.35% and showed the following trend: Mg30 < Mg90 < Mg120 (Fig. 1b). The amounts of Mg leached from the PIII-treated titanium were determined through inductively coupled plasma atomic emission spectroscopy (ICP-AES). The results indicated that the samples with longer PIII times released higher amounts of Mg. The concentration of Mg in the resulting solution for each group increased with the duration of immersion, as shown in Fig. 1c. The results of contact angles are displayed in Fig. 1d. The Mg PIII treatment did not change the hydropathy property of sample surfaces compared with the Ti surface.

### *In Vitro* Responses of Macrophages

Most of the cells in the control group were round and flat, whereas the cells in the Mg PIII-treated groups were more elongated and less flattened (Fig. 2a). There were no significant differences in cell numbers among groups, as shown in Fig. 2b. There were no statistically significant differences in CCK-8 results between the Mg PIII-treated groups and titanium groups, as shown in Fig. 2c, thus indicating that magnesium doping had no obvious toxic influence on the proliferation of macrophages.

The cells cultured on the surface of Mg PIII-treated titanium expressed less iNOS than that in cells cultured on the titanium control, and the amount decreased as the concentration of Mg on the samples increased (both day 1 and day 4 have similar patterns); in contrast, the expression of CD206 was increased (Fig. 3). The dot plots from a representative flow cytometry experiment are presented in Fig. 4a and b. The percentage of M2 cells expressing the surface marker CD206 showed the following trend: Ti < Mg30 < Mg90 < Mg120 (Fig. 4d). By contrast, the percentage of M1 cells expressing the surface marker C-C motif chemokine receptor 7 (CCR7) showed the following trend: Ti > Mg30 > Mg90 > Mg120 (Fig. 4c). The differences among the various groups were statistically significant, especially after 4 days of culture.

The TNF-α concentration was lower in the supernatants recovered from Mg PIII-treated titanium compared with the titanium control, but the only statistically significant difference on day 1 was between the Ti and Mg30 groups. However, the differences in TNF-α concentration became obvious after 4 days of culture, and the trend was as follows: Ti > Mg30 > Mg90 > Mg120 (Fig. 4e). The concentrations of IL-6 in the medium retrieved from Mg PIII-treated groups were also lower than that from cells grown on titanium, both on day 1 and on day 4 after the RAW cells were seeded (Fig. 4f). Higher levels of the anti-inflammatory cytokine IL-4 were found in the Mg PIII-treated groups than in the titanium control, and these differences were statistically significant both on day 1 and on day 4 (Fig. 4g). Another anti-inflammatory cytokine, IL-10, was found increased in RAW cells cultured on the Mg PIII-treated titanium on day 1 and day 4, compared with the titanium group. On day 4 the difference was more obvious, as shown in the following trend: Ti < Mg30  < Mg90 < Mg120 (Fig. 4h). Together, these results indicate that Mg PIII treatment induced the production of lower levels of pro-inflammatory cytokines but higher levels of anti-inflammatory cytokines, thus demonstrating a characteristic of M2 macrophage response.

The expression of CD86, a surface marker gene for the M1 phenotype, was down-regulated in the Mg PIII-treated groups (Fig. 5a), whereas the M2 marker gene CD163 was up-regulated (Fig. 5b). The gene expression levels of the two growth factors (BMP2 and VEGF, both of which promote tissue healing) produced by the RAW cells were markedly increased in the Mg PIII-treated groups compared with the control group (Fig. 5c,d).

The western blot bands are shown in Fig. 5e. The expression of NF-κB was down-regulated in cells grown on Mg PIII-treated titanium compared with the titanium control. The trend of NF-κB expression was as follows: Ti > Mg30 > Mg90 > Mg120 (Fig. 5f). In contrast, the expression of nuclear factor of kappa light polypeptide gene enhancer in B-cells inhibitor alpha (IκB-α) was up-regulated and showed the following trend: Ti < Mg30 < Mg90 < Mg120 (Fig. 5g). The original bands are shown in supplementary information.

### *In Vivo* Responses of Macrophages

As shown in Fig. 6, at 1 and 4 days after surgery, higher numbers of M2 macrophages were observed in the Mg PIII-treated groups compared with the titanium control, and lower numbers of M1 macrophages were observed. The total number of cells adhered to the samples increased significantly as the indwelling time increased.

A general view of the fibrous layer and infiltrated inflammatory cells surrounding the implanted samples was observed in the lower magnification images, and in the higher magnification images, iNOS- or CD206-positive cells were identified (Fig. 7). As depicted in Fig. 8, the fibrous layer thickness, the total cell number, and the number of iNOS-positive cells in the Mg PIII-treated groups were lower than for the titanium control (Ti > Mg30 > Mg90 > Mg120); in contrast, higher percentages of CD206-positive cells were observed in the Mg PIII-treated groups (Ti < Mg30 < Mg90 < Mg120). The trend was more apparent 7 days after implantation. The quantitative results were consistent with the general observation (Fig. 7).

Dot plots from a representative flow cytometry experiment are depicted in Fig. 9a and b. The statistical results are shown in Fig. 9c and d. The use of specific macrophage phenotypic markers showed that the inflammatory exudates collected from the air pouches implanted with Mg PIII-treated titanium elicited lower percentages of F4/80 and CCR7 double-positive cells (representing an M1 macrophage phenotype), compared with the titanium control (Ti > Mg30 > Mg90 > Mg120). In contrast, higher percentages of F4/80 and CD206 double-positive cells (representing an M2 macrophage phenotype) were identified in the exudates retrieved from Mg PIII-treated groups than the Ti group (Ti < Mg30 < Mg90 < Mg120). In total, the Mg PIII-treated titanium triggered more M2 macrophage phenotypes and fewer M1 macrophage phenotypes than the titanium control, and the differences became more significant with increasing Mg content, especially 4 days after surgery.

As shown in the significant results in Fig. 9e, the concentrations of TNF-α in the Mg PIII-treated groups were lower than those in the titanium control both at day 1 and at day 4. No differences were observed in the concentration of IL-6 between all groups at day 1. However, a lower concentration of IL-6 was detected in Mg PIII-treated groups at day 4, and the trend was as follows: Ti > Mg 30 > Mg90 > Mg120 (Fig. 9f). The anti-inflammatory cytokines IL-4 and IL-10 were increased in the exudates from the Mg PIII-treated samples at both day 1 and day 4. The difference was more apparent at day 4 and showed the following trend: Ti < Mg 30 < Mg90 < Mg120 (Fig. 9g and h). These data suggest that the Mg PIII-treated samples induced lower concentrations of inflammatory cytokines but higher concentrations of anti-inflammatory cytokines.

## Discussion

The homeostasis of the immune cell state is indispensable for tissue development, regeneration, and repair^19^. Trauma caused by indwelling of biomaterials initiates a series of immune responses that mobilize various types of immune cells into the wound site and activate host defence and tissue repair. Among these cells, macrophages have received considerable attention as modulators promoting better tissue remodelling outcomes. Regulation of macrophage state by surface modification of biomaterials is emerging as an innovative strategy to repair damaged tissues^6^. In this study, different amounts of magnesium were introduced onto the surface of titanium through plasma immersion ion implantation (Mg PIII). We found that doping with magnesium significantly regulates the polarization of macrophages (in this case, the murine cell line RAW 264.7) *in vitro* and *in vivo*. Specifically, the Mg PIII-treated titanium modulated macrophages towards the M2 phenotype, which promotes tissue healing, and reduced the host inflammatory response against the materials. The trend became more apparent as the concentration of Mg increased.

Changes in macrophage cell shape are thought to be related to polarization state. We found that the morphology of RAW 264.7 cells seeded on Mg PIII-treated groups appeared to be more elongated and less spread than in the titanium control. Although it is difficult to quantitatively describe differences along the continuous spectrum of macrophage characteristics, the immunostaining results clearly showed that the Mg PIII treatment up-regulated the M2 marker CD206 and down-regulated the M1 marker iNOS (Fig. 3). The expression of phenotypic markers revealed a significant difference between the groups, i.e., the Mg PIII-treated groups induced a higher percentage of CD206-positive M2 cells and a lower percentage of CCR7-positive M1 cells than did the titanium group (Fig. 4c,d). The changes in cytokine levels, as evaluated by ELISA, further confirmed the functional differences between the macrophage phenotypes. The cells on the Mg PIII-treated surfaces secreted higher concentrations of two anti-inflammatory cytokines, IL-4 and IL-10, and lower concentrations of two pro-inflammatory cytokines, TNF-α and IL-6 (Fig. 4e,f,g,h). The trend was more apparent with longer culture times. At the genetic level, Mg PIII-treated titanium also altered the expression of two specific markers of macrophage polarization, CD86 and CD163. Together, these data demonstrate that the Mg-PIII treated titanium induced higher numbers of M2 cells and lower numbers of M1 cells *in vitro*. In addition, gene expression levels of two growth factors, BMP2 and VEGF, were elevated in the Mg PIII-treated group. Those two factors are known to promote wound healing and bone formation. Thus, these findings indicated that the change in macrophage polarization state might be one of the mechanisms accounting for the osteogenic effect of Mg. The specific relationship between macrophage polariztion and osteogenesis may be an important area for future investigation.

NF-κB activation was reduced in Mg PIII groups and was accompanied by an increased level of IκB-α. This inhibitory effect of Mg on the NF-κB signalling pathway is consistent with results from previous studies^13^,^20^,^21^,^22^. This phenomenon might also be one of the mechanisms underlying the inhibitory effect of Mg PIII treatment on M1 macrophage differentiation^23^,^24^. L-type calcium channels, phosphoinositide 3-kinase/Akt and phosphoinositide 3-kinase β, δ, and γ are involved in the anti-inflammation effects of Mg^25^,^26^,^27^. The exact molecular mechanisms whereby Mg affects macrophage polarization and inflammation need to be investigated further.

In this study, we also investigated the immunomodulatory effects of Mg PIII treatment on macrophage phenotypic profile in a mouse air pouch model of inflammation *in vivo*. The air pouch model has been extensively used in other experiments in research on various types of inflammation because of its advantages of high sensitivity and convenience for analysis of features from histology to cytokine levels^28^,^29^. The immunofluorescence staining results of cells that had adhered to sample surfaces revealed that the Mg PIII-treated titanium induced more M2 cells and fewer M1 cells than did the titanium control. The histological analysis showed that the Mg PIII-treated titanium caused a significant decrease in the number of inflammatory cells recruited to the implant site, together with a higher percentage of M2 cells verified by immunohistochemistry. These results were further complemented by the quantitative assessment of macrophage profiles by flow cytometry and of the levels of cytokines present in the inflammatory exudates. Higher percentages of M2 macrophages with higher concentrations of anti-inflammatory cytokines (IL-4 and IL-10) and lower percentages of M1 macrophages with lower concentrations of pro-inflammatory cytokines (TNF-α and IL-6) were detected in the Mg PIII-treated groups than in the titanium group. The foreign body reaction, with encapsulation of the implanted medical device, is a major complication after implantation that impairs device function^6^. We found that the thickness of the fibrous capsule around the Mg PIII-treated samples was significantly decreased compared with that in the Ti control. This decrease might be one of the beneficial outcomes of modulating macrophages towards the M2 phenotype at the early stage of inflammation. This phenomenon might have been due to the limitation of the foreign body reaction. The time to modulate macrophages towards the M2 phenotype should also be taken into consideration, because macrophages play multiple roles in different stages of inflammation and tissue healing. The exact molecular mechanism is an important area for future investigation. In general, the data *in vivo* are consistent with the data *in vitro*, and together they demonstrate the immunomodulatory effects of Mg PIII-treated titanium on macrophage polarization.

Not only the chemistry of biomaterials but also physical cues, including material geometry, pore size and pore shape, may affect macrophage phenotype^30^. The similar topography among all sample surfaces observed by SEM excluded the influence of physical cues on the macrophage phenotype. The ICP-AES result indicated that the concentration of released magnesium ions increased with the extension of plasma immersion ion implantation time. The concentration of Mg ions detected by ICP-AES was at a very low level. The concentration might have been higher at the contact surface, but there is no way to test this possibility to date. By contrast, the concentration of Mg ions used for anti-inflammation effects in previous research has been relatively high level (60 mg/L or 2.5 mM). This concentration is known to be clinically effective but it is very close to the toxic dose^14^. The PIII technique provided a strategy for local delivery of Mg. The Mg PIII-treated titanium released magnesium ions locally at such a low level that hypermagnesaemia was not a concern. Interestingly, the degree of M2 polarization almost paralleled the increase in magnesium (Ti < Mg 30 < Mg90 < Mg120). The exceptions of CD163 and BMP2, with Mg30 inducing a higher level of gene expression, might have been due to the different sensitivities of different markers. This possibility may be an important area for future investigation. Moreover, the difference in timing between gene and protein expressions should be taken into consideration. The amount of Mg implanted on the titanium surface reached its peak level at 120 min of implantation, and there was no significant futher increase of Mg with increasing implantation time. Excessive concentrations of Mg ions may trigger detrimental inflammation, which is not beneficial to tissue healing^31^. Therefore, whether there is an optimal concentration of Mg ions to maximize M2 polarization requires further investigation.

## Conclusion

The responses of macrophages to titanium doped with Mg through the plasma immersion ion implantation (Mg PIII) technique were evaluated both *in vitro* and *in vivo*. Small amounts of Mg doping on a titanium surface facilitated the differentiation of an M2 anti-inflammatory, pro-tissue healing macrophage phenotype. This change contributed to the greater expression of the growth factors BMP2 and VEGF *in vitro* and less fibrous tissue formation *in vivo*. This immunomodulatory effect may be due to the suppression of the NF-κB signalling pathway. These results highlight the potential utility of Mg PIII treatment to elicit better outcomes after implantation by modulation of immunity.

## Materials and Methods

### Preparation of material

Magnesium was doped on titanium surfaces by using the cathodic arc sourced magnesium plasma immersion ion implantation (Mg PIII) technique. Commercial pure titanium (Cp Ti, Grade 2) was used as the substrate and control group. The titanium surface was pretreated in a 5 wt% oxalic acid solution at 100 °C for 2 h and was ultrasonically cleaned in distilled water. The Mg PIII-treated groups were designated Mg30 (PIII at 30 kV for 30 min), Mg90 (PIII at 30 kV for 90 min), and Mg120 (PIII at 30 kV for 120 min). The detailed doping procedures were as previously described^32^,^33^. Both sides of each sample were doped with magnesium.

### Material characterization

SEM (S-3400, HITACHI, Japan) was used to examine the surface morphologies of the four groups. The surface chemical composition was examined with XPS (AXIS UltraDLD, Kratos, Japan). The release kinetics of Mg were evaluated by using a previously described method^17^. In brief, the samples (2 cm squares) were immersed in 10 mL phosphate buffer solution (PBS) for various durations at 37 °C without agitation. The resultant solutions were analysed by using ICP-AES. The surface wettability of the samples was evaluated on the basis of contact angle measurements (Automatic Contact Angle Meter Model SL200B, Solon, China). Data were collected after a 2 μL deionized water droplet was dropped onto the sample surface and stabilized at room temperature. Three samples in each group were tested for statistical analysis.

### *In vitro* study

The RAW 264.7 (RAW) murine-derived macrophage cell line was obtained from the Cell Bank of the Chinese Academy of Science and maintained in Dulbecco’s modified Eagle’s medium (DMEM; HyClone) supplemented with 10% heat-inactivated foetal bovine serum (FBS, Gibco) and 1% penicillin/streptomycin (Gibco) at 37 °C in a humidified atmosphere of 5% CO2. The culture medium was exchanged every 48 h. The growing cells were passaged at approximately 80% confluence by scraping, and only early passages (p3-5) were used in the study.

To observe the cell morphology, cells (1 × 10^5 ^cells/well) were cultured on 24-well plates with different samples. The samples were washed with PBS and fixed with 2.5% glutaraldehyde at 4 °C for 2 h. Further dehydration was conducted with ethanol at different concentrations (30, 50, 75, 90, 95, and 100 v/v%) for 10 min each. Then, the cells were freeze-dried, sputter-coated with platinum, and observed through SEM.

To evaluate cell proliferation, cells (1 × 10^5 ^cells/well) were seeded onto different samples (10 mm × 10 mm). Cell number on the surface was counted on the basis of five randomly separated horizons. After 1 and 4 days of culture, 50 μL CCK-8 (Dojindo, Japan) solution and 450 μL culture medium were added to each well, and the cells were further incubated for 4 h. Finally, the absorbance was measured with a microplate reader at a wavelength of 450 nm after addition of 100 μL of each incubated solution to a 96-well plate.

Immunofluorescence staining assays were carried out to qualitatively analyse the expressions levels of iNOS (M1 marker) and CD206 (M2 marker). RAW cells (1 × 10^5 ^cells/well) were seeded onto different samples (10 mm × 10 mm). After being cultured for 1 and 4 days, the cells were fixed with 4% paraformaldehyde for 15 min at room temperature and then washed 3 times in PBS containing 0.1% Triton-X to permeabilize them. The cells were then blocked with 10% FBS for 30 min in PBS. Primary antibodies for iNOS (Novus Biologicals) and CD206 (AbCam) were incubated with the cells at 1:50 in PBS with 1% FBS and at 4 °C overnight. Secondary antibodies (AbCam) donkey anti-rabbit Alexa Fluor 488 (1:200), Donkey Anti-Mouse Alexa Fluor 594 (1:200) were incubated with the cells at room temperature for 2 h. DAPI was used to stain the cell nuclei. Images were obtained using a fluorescence microscope (Leica).

Flow cytometry analysis was carried out to quantitatively analyse the expression of CCR7 (M1 marker) and CD206 (M2 marker). In total, 5 × 10^5^ cells were seeded onto different samples (20 mm × 20 mm). After 1 and 4 days of culture, the cells were trypsinized and scraped from the sample surfaces, centrifuged and resuspended in 1% bovine serum albumin (BSA) for 30 min at ambient temperature to block non-specific antigens. The cells were then incubated with fluorescein isothiocyanate (FITC)-conjugated anti-mouse F4/80, allophycocyanin (APC) -conjugated CCR7 and phycoerythrin (PE) -conjugated CD206 for 1 h in the dark at ambient temperature with a final volume of 100 μL. FITC-conjugated rat IgG2a,κ, APC-conjugated rat IgG2a,κ and PE-conjugated rat IgG2a,κ were used as isotype controls. All flow cytometry antibodies were from eBioscience. After being washed twice in 1% BSA, the cells were resuspended in 1% BSA and analysed with a Guava flow cytometer (Millipore, USA); 5, 000 cells were analysed in each test. Data were analysed in guavaSoft 3.1.1 software.

The levels of relevant cytokines were measured. Cytokine production was assessed using ELISA. After 1 and 4 days of culture, the culture medium was aspirated and centrifuged, and the supernatant was used for analyses. The concentrations of TNF-α, IL-4, IL-6, IL-10 were determined using ELISA kits (Anogen, Canada), following the manufacturer’s instructions.

PCR was carried out to evaluate the gene expression of the specific macrophage surface markers CD86 and CD163, representing M1 and M2, respectively, and the growth factors BMP2 and VEGF. RAW cells were seeded onto different samples (20 mm × 20 mm) at a density of 5 × 10^5^ cells per sample and cultured for 4 days. The culture medium was removed. After cells were washed twice with PBS, the RNA was extracted using TRIzol reagent (Invitrogen). Three hundred nanograms of total RNA was used to synthesize complementary DNA using a PrimeScript RT Reagent Kit (Takara) by following the manufacturer’s instructions. SYBR Premix Ex TaqII (Takara) was used for detection, and expression levels of the target mRNAs were assayed on a Bio-Rad C1000. The mean threshold cycle (Ct) value of the housekeeping gene GAPDH was used to normalize the target genes. The **2**^**−ΔΔCt**^ method was used to compare the mRNA expression levels between different groups. Table 1 shows the primers for the target genes.

A western blot was carried out to determine the NF-κB signalling pathway-related protein expression of NF-κB and IκB-α. Fifteen micrograms of protein from each sample was resolved by sodium dodecyl sulfate-polyacrylamide gel electrophoresis (SDS-PAGE) and transferred to nitrocellulose membranes. The membranes were blocked in 5% non-fat dry milk in TBS-T buffer (25 mM Tris-HCl, 140 mM NaCl, 0.1% Tween 20, pH 7.5) for 1 h and incubated with primary antibodies against NF-κB (1:1000, Abcam), IκB-α (1:1000, Cell Signalling Technology) and α-tubulin (1:5000, Abcam) at 4 °C overnight. After being washed three times in TBS-Tween buffer, the membrane was incubated with horseradish peroxidase-conjugated secondary antibodies for 1 h at room temperature. The protein bands were visualized using ECL-plus chemiluminescence (Amersham, USA) according to the manufacturer’s instructions. The relative intensity of protein bands was quantified using Image-Pro Plus software.

### *In vivo* study

Animal care and use were in accordance with the guidelines established by the Administration of Affair Concerning Laboratory Animals for Shanghai Jiao Tong University, the National Institutes of Health Guide for Care and Use of Laboratory Animals (GB14925-2010) and the Regulations for the Administration of Affairs Concerning Experimental Animals (China, 2014). All animal experiments described in this study were approved by the Animal Care and Experiment Committee of Shanghai Sixth People’s Hospital affiliated with Shanghai Jiao Tong University. Air pouches were generated according to the method of Sedgwick *et al*.^34^ For each experimental group, 6 male C57BL/6 mice, 8 weeks old, were used. All the mice were injected subcutaneously in the dorsal area with 5 mL sterile air that caused the formation of an air pouch. A second injection of the air pouch was performed 5 days later with 3 mL sterile air. One day after the second injection, the mice were anaesthetized via intraperitoneal injection of chloral hydrate (350 mg/kg). The skin covering the air pouch area was shaved and sterilized. A surgical incision was made, one of the samples (1 cm squares, both sides doped with Mg) was implanted into the air pouch and the incision was sutured.

*In vivo* immunocytochemistry analysis was carried out to determine the expression levels of specific markers for M1 (iNOS) and M2 (CD206) macrophages. The mice were anaesthetized and sacrificed 1 and 4 days after surgery. The samples were carefully removed from the pouches and fixed with 4% paraformaldehyde in PBS for 30 min. Then, the samples were washed in PBS three times to remove paraformaldehyde. Non-specific antigens of the cells attached to the surface of the samples were blocked with 10% FBS for 30 min in PBS. Primary antibodies for iNOS (Novus Biologicals) and CD206 (AbCam) were incubated with the cells at 1:50 in PBS with 1% FBS and at 4 °C overnight. Secondary antibodies (AbCam) donkey anti-rabbit Alexa Fluor 488 (1:200), Donkey Anti-Mouse Alexa Fluor 594 (1:200) were incubated with the cells at room temperature for 2 h, as previously described.

Histological analysis was carried out for morphological observation and specific macrophage phenotype identification. The tissues surrounding the samples were retrieved at day 4 and day 7 after the surgery. The tissues were fixed in 10% neutral buffered formalin, embedded in paraffin and cut into 5 μm sections. Then, the sections were stained with haematoxylin-eosin (HE) and immunohistochemistry. 3% hydrogen peroxide (Sigma-Aldrich) in 50% methanol was used to block endogenous peroxidase for 5 min and 3% BSA was used to block non-specific antigens. Subsequently, a primary antibody against iNOS (Novus Biologicals) at a 1:20 dilution or CD206 (AbCam) at a 1:50 dilution was incubated with the tissue sections at 4 °C overnight. An undiluted horseradish peroxidase (HRP)-conjugated secondary antibody was applied, and diaminobenzidine (DAB) substrate was used to stain the sections. The cell nuclei were stained with haematoxylin, and the results were analysed with a light microscope. Image-Pro Plus software was used to quantitatively analyse the thickness of fibrous layer, the number of infiltrated cells and the percentage of iNOS-positive (M1) or CD206-positive (M2) cells.

*In vivo* flow cytometry analysis was carried out to determine the expression levels of two specific markers, CCR7 (M1) and CD206 (M2). The mice were anaesthetized and sacrificed 1 and 4 days after implantation. After the mice were sacrificed, the inflammatory exudates were harvested by washing the air pouch cavities with 2 mL of PBS, and this was followed by recovery of the lavage fluid. The exudates were filtered through 40 μm nylon mesh (BD Biosciences) to remove cell clumps and centrifuged at 1200 rpm for 5 min at 4 °C. Supernatants were discarded, and cell pellets were resuspended in 1 mL 1% BSA/PBS. The cell suspensions were preincubated for 30 min at ambient temperature to block non-specific antigens. The cells were stained with the same antibodies as were used *in vitro*. After two washes in 1% BSA, the cells were resuspended in 1% BSA and analysed with a Guava flow cytometer (Millipore, USA). Data were analysed as previously described.

Cytokine analysis of the exudates was carried out. The exudates were centrifuged at 2500 rpm for 10 min. The concentrations of IL-4, IL-6, IL-10, TNF-α were measured using ELISA kits (Anogen, Canada), following the manufacturer’s instructions.

### Statistical analysis

All statistical analyses were performed using the SPSS 18.0 software (SPSS, Chicago, IL). All data are shown as the means ± standard deviation (SD). The data were analysed using one-way ANOVA followed by Tukey’s post hoc test. The level of significance was set to P < 0.05.

## Additional Information

**How to cite this article**: Li, B. *et al. In vitro* and *in vivo* responses of macrophages to magnesium-doped titanium. *Sci. Rep.* **7**, 42707; doi: 10.1038/srep42707 (2017).

**Publisher's note:** Springer Nature remains neutral with regard to jurisdictional claims in published maps and institutional affiliations.

## Supplementary Material

Supplementary Information

## Figures and Tables

**Figure 1:** (**a**) Scanning electron microscopy (SEM) images of titanium (Ti) and magnesium plasma immersion ion implantation (Mg PIII)-treated titanium with different doping time (Mg30, Mg90, Mg120), (**b**) X-ray photoelectron spectroscopy (XPS) spectra, (**c**) Mg concentrations released from Mg PIII-treated titanium at days 7, 14, 21 and 28, (**d**) Water contact angles of the samples. (Statistically significant difference: *p < 0.05; **p < 0.01; triplicate).

**Figure 2:** (**a**) Morphology of RAW 264.7 cells on various surfaces, as determined by SEM at day 1 and day 4, (**b**) RAW 264.7 cell number on the surface, (**c**) Cell proliferation evaluated with a Cell Counting Kit-8 (CCK-8). (Statistically significant difference: *p < 0.05; **p < 0.01; triplicate).

**Figure 3:** Images of immunofluorescent staining of the RAW cells adhered to various surfaces. iNOS (green fluorophore) indicates M1 macrophages; CD206 (red fluorophore) indicates M2 macrophages; nuclei are stained with DAPI (blue fluorophore); scale bar: 100 μm. (iNOS: inducible nitric oxide synthase; CD206: cluster of differentiation 206; DAPI: 4′,6-diamidino-2-phenylindole).

**Figure 4:** Expression of cell surface markers on RAW cells, as determined by flow cytometry; cytokines secreted by RAW cells on various surfaces, as determined by enzyme-linked immunosorbent assay (ELISA). Representative dot plots showing: (**a**) F4/80 and CCR7 double staining, (**b**) F4/80 and CD206 double staining, (**c**) Percentage of F4/80 and CCR7 double positive cells (M1), (**d**) Percentage of F4/80 and CD206 double positive cells (M2). Cytokine production: (**e**) TNF-α, (**f**) IL-6, (**g**) IL-4, (**h**) IL-10. (Statistically significant difference: *p < 0.05; **p < 0.01; triplicate). (F4/80: mouse epidermal growth factor-like module-containing mucin-like hormone receptor-like 1; CCR7: C-C motif chemokine receptor type 7).

**Figure 5:** Relative mRNA expression levels of macrophage polarization markers and growth factors: (**a**) CD86, (**b**) CD163, (**c**) BMP2, (**d**) VEGF. (**e**) Western blot assay of the NF-κB signalling pathway-related proteins NF-κB and IκB-α, (**f**,**g**) Statistical results of relative protein bands intensity. (Statistically significant difference: *p < 0.05; **p < 0.01; triplicate). (BMP2: bone morphogenetic protein 2; VEGF: vascular endothelial growth factor; NF-κB: nuclear factor κB; IκB-α: nuclear factor of kappa light polypeptide gene enhancer in B-cells inhibitor alpha).

**Figure 6:** Immunofluorescence images for iNOS (M1 phenotype, in green) and CD206 (M2 phenotype, in red) markers in adherent macrophages on various surfaces 1 and 4 days after surgery; nuclei stained with DAPI (in blue); scale bar: 50 μm.

**Figure 7:** Haematoxylin-eosin (HE) and immunohistochemistry (iNOS and CD206) analysis of tissues adjacent to the indwelling samples at day 4 (**a**) and day 7 (**b**). Blue arrows: fibrous layer. Yellow rectangle: indicate the location of implants. Scale bar: 50 μm.

**Figure 8:** Quantitative analysis of (**a**) fibrous layerthickness, (**b**) number of infiltrated cells, (**c**) iNOS-positive cells (M1) and (**d**) CD206-positive cells (M2). (Statistically significant difference: *p < 0.05; **p < 0.01; triplicate).

**Figure 9:** Flow cytometry analysis of cell surface markers on macrophages harvested from the mouse air pouches; cytokines in the air-pouch exudates, as determined by ELISA. Representative dot plots showing: (**a**) forward scatter (FSC) and side scatter (SSC), (**b**) expression of CCR7 (M1) and CD206 (M2) antigens. Macrophages were gated by F4/80-positive. (**c**) Percentage of F4/80 and CCR7 double-positive cells (M1), (**d**) Percentage of F4/80 and CD206 double-positive cells (M2). Cytokine production: (**e**) TNF-α, (**f**) IL-6, (**g**) IL-4, (**h**) IL-10. (Statistically significant difference: *p < 0.05; **p < 0.01; triplicate).

**Table 1:** Primers for RT-PCR.

Gene	Primer sequences (F, forward; R, reverse; 5′−3′)
CD86	F: TGC TCA TCA TTG TAT GTC AC
	R: GTC TCT CTG TCA GCG TTA CT
CD163	F: TCA GCG ACT TAC AGT TTC CTC
	R: GCC TTT GAA TCC ATC TCT TG
BMP2	F: TAC CTG TCC TAC TCA CCG AT
	R: CTT CAC TGC CTT GTC AAC AT
VEGF	F: GCA AGA GAA GAC ACG GTG GT
	R: CAG GAG GTG GGG TAA GGA G
GAPDH	F: AAA TGG TGA AGG TCG GTG TG
	R: AGG TCA ATG AAG GGG TCG TT
